# UXT at the crossroads of cell death, immunity and neurodegenerative diseases

**DOI:** 10.3389/fonc.2023.1179947

**Published:** 2023-04-19

**Authors:** Pengzhe Han, Shaojian Mo, Zhengwang Wang, Jiale Xu, Xifeng Fu, Yanzhang Tian

**Affiliations:** ^1^ Third Hospital of Shanxi Medical University, Shanxi Bethune Hospital, Shanxi Academy of Medical Sciences Tongji Shanxi Hospital, Taiyuan, China; ^2^ Department of Biliary and Pancreatic Surgery, Shanxi Bethune Hospital, Shanxi Academy of Medical Sciences, Tongji Shanxi Hospital, Taiyuan, China

**Keywords:** UXT, apoptosis, immunity, neurodegenerative disease, autophagy

## Abstract

*The ubiquitous expressed transcript (UXT)*, a member of the prefoldin-like protein family, modulates regulated cell death (RCD) such as apoptosis and autophagy-mediated cell death through nuclear factor-κB (NF-κB), tumor necrosis factor-α (TNF-α), P53, P62, and methylation, and is involved in the regulation of cell metabolism, thereby affecting tumor progression. UXT also maintains immune homeostasis and reduces proteotoxicity in neuro-degenerative diseases through selective autophagy and molecular chaperones. Herein, we review and further elucidate the mechanisms by which UXT affects the regulation of cell death, maintenance of immune homeostasis, and neurodegenerative diseases and discuss the possible UXT involvement in the regulation of ferroptosis and immunogenic cell death, and targeting it to improve cancer treatment outcomes by regulating cell death and immune surveillance.

## 1 Introduction

*The ubiquitous expressed transcript (UXT)* gene is located at the Xp11.23–p11.22 locus, a region of strong biological significance that is affected by X gene inactivation. When retrieved from the National Center for Biotechnology Information (NCBI, https://www.ncbi.nlm.nih.gov/gene) UXT is also known as *STAP1* and *ART-27*. Recent studies have revealed that *UXT* plays an important role in cellular transformation and gene transcription by regulating the androgen receptor (AR), GATA4, nuclear factor-κB (NF-κB), and EVI1activities as cofactors (1–5). UXT is upregulated in various tumor tissues, including colorectal cancer (6), sarcoma (5), breast cancer (7, 8), and dedifferentiated skull-base chordomas (9). Therefore, UXT is considered a proto-oncogene in human cancers. UXT is downregulated in prostate cancer tissues, and its overexpression has been reported to inhibit prostate cancer cell growth (10–12). UXT may promote or suppress tumorigenesis depending on the tumor type and microenvironment (13).

Previous research has confirmed that: ​UXT contains two mRNA splicing variants that produce two UXT isoforms, UXT-V1 and UXT-V2, respectively. These two isoforms differ in their subcellular localization and actions, with the UXT-V2 protein mainly distributed in the nucleus and the UXT-V1 protein mainly distributed in the cytoplasm (14). At the same time, the expression of UXT-V1 is lower than that of UXT-V2. Some of the studies did not specifically state the isoforms; for those studies, “UXT” is used in this review.

**​**Cell death is an important mechanism for maintaining the functional homeostasis of cells or organs (15). In the treatment of tumors, targeting or inducing tumor cell death is also the pathway of choice for most non-surgical treatment modalities for tumors, and therefore the study of the mechanisms regulating cell death is crucial (16). However, tumor cells are resistant to cell death. This involves activation of anti-apoptotic proteins, cellular autophagy, and epigenetic mechanisms. Chemotherapy resistance caused by them is a difficult problem in most cancer treatments (17). As the research of tumor treatment has advanced, the clinical treatment of tumor has entered the era of precision medicine. Targeted therapy and immunotherapy are gradually gaining attention (18). Cell death releases substances such as damage associated molecular patterns, ATP, DNA and inflammatory factors, which activate anti-tumor immune response. Thus, cell death induces different levels of immune response (19). Amyotrophic lateral sclerosis (ALS) is one of the neurodegenerative diseases. ALS is associated with neuroinflammation, immune response, and dysfunction due to neuronal death (20, 21).

There are some contradictory views among studies on the role of UXT. First, UXT-V2 can inhibit TNF-α-induced apoptosis by upregulating the expression of anti-apoptotic genes in the NF-κB signaling pathway (2). In addition, UXT can also inhibit P53 activity through murine double minute X (MDMX) or epigenetic mechanisms, thereby suppressing apoptosis (5, 22). However, UXT-V2 can also interact with sterile α and HEAT armadillo motif-containing protein (SARM) in mitochondria to promote apoptosis (23). Second, UXT can promote P62-mediated selective autophagy (24, 25). However, when UXT is downregulated, it can promote autophagy by decreasing mTOR activity or promoting autophagy lysosome formation (26, 27). Third, UXT-V1 knockdown inhibits type I IFN expression (28), and UXT-V2 is phosphorylated to impair the activation of NF-κB signaling pathway and attenuate host cell antiviral immune responses (29). However, UXT can inhibit the expression of type I IFN through the cGAMP-STING signaling pathway (25). Therefore, there is an urgent need to evaluate the role of UXT in different diseases. To this end, we present a comprehensive review on the different ways in which UXT regulates cell death and the progress of UXT research in immune regulation and neurodegenerative diseases based on the perspectives of cell death and immunity. We also discuss the possibility of UXT involvement in ferroptosis, immunogenic cell death, the improvement of the tumor immune microenvironment and immune response, and the regulation of neuro-degenerative disease progression. We reveal possible research trends and indicate some suggestions for future research.

## 2 The origin and degradation of UXT

The *UXT* gene encodes a protein of approximately 18 kDa and is widely expressed in human and mouse tissues (30). UXT is a member of the alpha-like prefoldin protein family that exhibits alpha-helical properties and has two isoforms, both of which are derived from the same chromosome. UXT is distributed in the nucleus, cytoplasm, and mitochondria. UXT-V2 is the shorter isoform, consisting of 157 amino acids, while UXT-V1 has 12 more amino acids (169 amino acids) at its N-terminal end compared with UXT-V2. These are called MVFPLPTPQEPI motif (31), which can bind to TRAF2 to mediate the TNFR1 apoptosis pathway, which is unique to UXT-V1. The UXT-V1 plasmid also generates the UXT-V2 isoform through translation at the second methionine of codon 13 (ATG2) (14). The subcellular localization of UXT correlates with the cell cycle. UXT binds to γ-microtubule proteins, suggesting that UXT is a centrosome component, and that its overexpression disrupts centrosome structure (11). UXT is also involved in mitosis and germ cell meiosis (32), and is essential for cell viability, with insufficient expression in cells leading to cell death (33).

Both UXT-V1 and UXT-V2 can be ubiquitinated. Both tumor suppressor protein LOX-PP and E3 ubiquitin ligase SCF (Fbxo7) can induce UXT-V2 ubiquitination and proteasome degradation (7, 14). UXT-V2 is highly expressed in breast cancer tissue, where it can inhibit ER activity. Endocrine therapy for ER-negative breast cancer is known to be less effective, and endocrine therapy for ER-positive patients also faces the dilemma of drug resistance and reduced sensitivity. This provides a new perspective on improving the poor response to endocrine therapy and resistance in breast cancer patients. E3 ubiquitin ligase SCF (Fbxo7) mediated ubiquitination of UXT-V1, but the cell abundance of UXT-V1 did not change significantly (14). The MVFPLPTPEPI motif at the N-terminal of UXT-V1 probably does not mediate ubiquitin binding of UXT-V1 to SCF (Fbxo7), at least not primarily. Although UXT-V1 is a short half-life protein, the regulation of its degradation remains unclear.

## 3 Apoptosis: one of the cell death pathways

Cell death is the end of cellular life. With the accumulation of experimental data in recent decades, multiple forms of cell death have been identified that are interconnected and complementary *via* mechanisms that regulate cellular homeostasis in living organisms. The Nomenclature Committee on Cell Death (NCCD) classifies cell death into regulatory cell death (RCD) and accidental cell death (ACD) based on environmental and environmental factors (34). RCD includes apoptosis (both endogenous and exogenous), necrosis, pyroptosis, ferroptosis, and autophagy-dependent cell death.

Targeting apoptotic pathways in tumor cells is a promising anticancer strategy (35, 36). Indeed, apoptosis, which is classified into either endogenous or exogenous based on the activating pathways, can be activated by cellular stress, DNA damage, and immune surveillance pathways. The key step in the endogenous apoptosis pathway is an altered mitochondrial outer membrane permeability (MOMP) with the release of Cyto-chrome c from the mitochondria into the cell matrix; this is accompanied by the dysregulation of the B-cell lymphoma 2 (BCL-2) family such as BH3-only protein, which activates caspase-9-mediated apoptosis (34). Conversely, exogenous apoptosis is mediated by Fas, TNF receptor 1 (TNFR1), death receptor (DR) 4, and DR5 membrane protein receptors, which correspond to Fas ligand (FasL), TNF, or TNF-related apoptosis-inducing ligand (TRAIL) proteins, respectively, and subsequently cause apoptosis through the recruitment of Fas-associated death domain (FADD) and caspase-8, which further activates the cascade of cysteine activation and BID cleavage (34). BID serves as the “link” between endogenous and exogenous apoptosis, and is positively regulated by p53 at the transcriptional level (37), which can transmit the signal to the mitochondria and trigger a stronger apoptotic signal.

### 3.1 UXT and mitochondria

Mitochondria provide energy for cells through diverse metabolic functions and play a central role in apoptosis. Recent studies have shown that mitochondria also play a novel role as pro-inflammatory signaling hubs in some types of cell death, such as necrosis, ferroptosis, and pyroptosis (38). The distribution of mitochondria is regulated by the cytoskeleton, and mitochondrial aggregation in the perinuclear region is considered a feature of cell death.

UXT interacts with leucine-rich pentatricopeptide repeat containing protein (LRPPRC) through the SEC1 structural domain and participates in the LRPPRC complex by acting as a bridge between the LRPPRC actin-based cytoarchitecture and potential transcriptional complexes. The LRPPRC complex participates in the integration of cytoskeletal actin and microtubule networks, including vesicular transport, nucleocytoplasmic shuttling, nuclear chromosome remodeling, and transcriptional control (39). Subsequently, it was shown that UXT, as one of the subunits of the LRPPRC complex, acts through the microtubule (MT) cytoskeleton, where normal cells need adenosine triphosphate the most and thus influence mitochondrial distribution, and localizes mitochondria at the key functional sites of chromosome remodeling where errors trigger mitochondria-mediated cell death (40). Elevated levels of UXT may promote progressive mitochondrial aggregation and cell death through the association of UXT with LRPPRC (41). In recent years, several studies have investigated the influence of UXT on the cytoskeleton and its involvement in mitochondrial distribution. Previously, UXT was thought to affect mitochondrial distribution through LRPPRC. There is a lack of strong evidence on whether UXT affects mitochondrial repositioning through the cytoskeleton and the causal mechanistic studies of this in relation to cell death. Both UXT-V1 and UXT-V2 have been shown to interact with SARM in monocyte mitochondria, as observed under lipopolysaccharide (LPS) and polyinosinic:polycytidylic acid (poly I:C) simulated infection conditions (23). The interaction of UXT-V2 with SARM in the mitochondria increases SARM-induced exogenous apoptosis by increasing caspase-8 activity and mitochondrial membrane potential depolarization. In contrast, the interaction between UXT-V1 and SARM decreased caspase-8 activity and inhibited apoptosis.

The shift in mitochondrial membrane potential can regulate the release of apoptotic factors and mitochondrial membrane permeability (42); therefore, mitochondrial membrane potential plays an important role in apoptosis (43). Future studies should investigate how UXT acts through the mitochondria to affect apoptosis or other death pathways.

### 3.2 UXT and the NF-κB signaling pathway

The NF-κB family is composed of B cell-specific transcription factors that include c-REL, RelA (p65), RelB, NF-κB2 (p100/p52), NF-κB1 (p105/p50), and five DNA-binding proteins that bind to form homo- or heterodimers, which regulate gene transcription. When NF-κB is not activated in the cytoplasm, it binds to its specific repressor protein, IκB. When infection and stress damage occur in the body, TNF and interleukin-1 (IL-1) activate the IκB kinase (IKK) complex, trigger NF-κB translocation, activate the NF-κB signaling pathway, and regulate the transcription of target genes. NF-κB regulates innate and adaptive immune responses and modulates cell proliferation and apoptosis. NF-κB signaling pathways are involved in the development of cancer, diabetes, immune disorders, acquired immunodeficiency syndrome, COVID-19, and other diseases through their regulatory roles in inflammation, tumors, and immunity (44, 45). TNF is a pleiotropic cytokine belonging to the TNF superfamily. By binding to its cognate receptor, TNF-R1, it induces a signaling cascade that can lead to the upregulation of pro-inflammatory genes or cell death. TNF signaling is determined by the activity of two distinct spatiotemporal complexes: the TNF-R1 binding complex (complex-I), which drives NF-κB activation and the inflammatory response, and the secondary complex (complex-II), which can trigger cell death (46).

In prostate cancer cells, UXT-V2 acts as a transcriptional cofactor that interacts with P65 through the intact Rel homology structural domain (RHD) in response to TNF-α stimulation. UXT-V2 is passively recruited to NF-κB enhancers and functions as a nuclear chaperone to tightly regulate NF-κB target gene expression in the nucleus. Reduction in endogenous UXT-V2 significantly increases the propensity for TNF-α-induced apoptosis (2). The authors also found that in UXT-V1 knockdown cells, TNF-α synergistically activated caspase-8 and poly-ADP ribose polymerase (PARP), significantly promoting apoptosis, and the cells were highly sensitive to TNF-α induced apoptosis. To be specific, UXT-V1 in the cytoplasm blocked the recruitment of FADD by TRAF2 and inhibited the formation of complex - II(FADD-RIP-TRADD) through the N-terminal 12-amino acid motif-targeting complex -I (TRAF2-RIP-TRADD). Therefore, UXT-V1 inhibits TNF-α induced apoptosis by blocking the recruitment of the death receptor TNFR1 adaptor protein (31). The UXT is not controlled by the NF-κB signal path. The regulation of complex- II by UXT-V1 and the regulation of nuclear events in NF-κB signaling pathway by UXT-V2 clarified the differences between the two isoforms of UXT, enriched the mechanism of action of UXT, provided direct evidence of UXT and cell death, and also hinted at the possibility of UXT participating in the regulation of tumor, inflammation and immunity through the NF-κB signaling pathway. Interestingly, there appears to be some contradiction between this and Sethurathinam’s (23) findings. They proposed that UXT-V2 interacts with SARM in the mitochondria of monocytes to promote apoptosis, which UXT-V1 inhibits. UXT-V2 is mainly found in the nucleus, cytoplasm, and mitochondria. But most of it is in the nucleus. In addition to the differences between the cells themselves, different subcellular localization may involve different mechanisms, which does not rule out the possibility that they occur simultaneously.

The mechanism underlying the selective activation of the NF-κB signaling pathway by UXT is not fully understood. In COS-7 cells, LRP16 interacts with ART-27 and AR in an androgen-independent manner and participates in AR transactivation (47). Furthermore, LRP16, as an interacting factor of UXT, could be integrated into the NF-κB transcriptional enhancer in the nucleus to participate in the regulation of NF-κB. Meanwhile, increased TNF-α + cycloheximide (CHX)-induced apoptosis was observed in cells with downregulated LRP16 expression. Downregulation of LRP16 also increased cell sensitivity to TNF-α-induced apoptosis; the anti-apoptotic proteins X-linked inhibitor of apoptosis protein (XIAP) and FLICE-inhibitory protein (FLIP) were blocked (48). The mechanism of the interaction between UXT and LRP16 in cell death, such as apoptosis, has not been further investigated. In addition, UXT interacts specifically with the EZH1-SUZ12 complex to regulate the activation of NF-κB targets. EZH1and UXT knockdown significantly increased the percentage of apoptotic cells and the sensitivity of cells to apoptosis. The mechanism may be that EZH1 and UXT can regulate TNF and two induced anti-apoptosis genes, *BIRC2* (coding cIAP1) and *BIRC3* (coding cIAP2) (49). Therefore, UXT-V2 may co-regulate the nuclear events of NF-κB with LRP-16 and EZH1 (**Figure 1**).

**Figure 1:** UXT and NF-κB signaling pathway: When TNF-α binds to TNFR1 and UXT-V1 binds to TRAF2, apoptosis is inhibited by inhibiting the formation of complex- II by inhibiting FADD recruitment. UXT-V1 binds to the SARM on the mitochondrial membrane and inhibits the activity of casepase8, thereby inhibiting cell apoptosis. UXT-V2 binds to SARM up-regulating the activity of casepase8 and promoting apoptosis. UXT-V2 acts as an NF-κB enhancer to regulate the transcription of downstream genes in the NF-κB signaling pathway. EZH1 and LRP-16 participate in the composition of the NF-κB enhanceosome.

### 3.3 UXT and the P53 signaling pathway

*P53*, also known as *TP53*, has tumor-suppressive effects. In normal cells, P53 binds to its inhibitors, mouse double minute 2 homolog (MDM2) and MDMX, and maintains low levels of activity. When activated in the presence of hypoxia, DNA damage, and stress, P53 induces apoptosis, cellular senescence, and cell cycle arrest. *P53* regulates energy metabolism, inflammation, and epithelial-mesenchymal transition and plays a central role in DNA damage repair. Importantly, *P53* can be mutated in various tumors (50, 51). The P53 pathway plays various roles in cell death, including apoptosis (52), autophagy (53), pyroptosis (54), necrosis (55), and ferroptosis (56). This may involve complex crosstalk with the NF-κB pathway (57).

Kyoto Encyclopedia of Genes and Genomes (KEGG) and gene ontology (GO) analyses revealed that genes differentially expressed before and after *UXT* knockdown in HCT116 cells were associated with the P53 pathway (49), which suggests a relationship between UXT and the P53 signaling pathway in tumors. The authors also confirmed in human osteosarcoma cells that UXT-V2 inhibits P53 activity by binding to MDMX, which further leads to a selective increase in NF-κB activity. This up-regulates the expression of hypoxia-inducible factor-1α (HIF-1α), which in turn significantly increases the expression of glycolytic genes, such as *glucose transporter (GLUT)-1/3, hexokinase (HK)-2/3, lactate dehydrogenase A (LDHA)*, and *enolase (ENO)*, promoting glycolysis (5). This shift confers a proliferation and survival advantage to tumor cells. The authors also demonstrated that UXT-V2 affects NF-κB activity by increasing the nuclear localization of P65.

In solid tumors, hypoxia is a pervasive growth environment in tumor tissue and is progressively exacerbated by reduced vascularity in the tissue. The Warburg effect is a metabolic signature in which tumor cells rapidly break down glucose and glutamine through glycolysis while activating the expression of key enzymes to provide energy (58). This imparts a variety of properties, such as cellular resistance to death. Researchers have found that breast cancer cells exhibit increased anti-apoptotic properties when aerobic glycolysis is enhanced, while inhibition of HIF-1α inhibits aerobic glycolysis, reduces resistance to apoptosis, and promotes apoptosis (59). UXT-V2 is up-regulated in breast cancer tissues and cell lines, and down-regulates maternal expression 3 (MEG3) by binding to DNMT3B, thereby inhibiting the P53 signaling pathway (22).UXT-V2 also inhibits apoptosis and promotes the proliferation, migration, and invasion of breast cancer cells through its negative regulation of the P53 signaling pathway (22). This provides direct evidence that UXT modulates apoptosis *via* the P53 signaling pathway (**Figure 2**).

**Figure 2:** UXT and the P53 signaling pathway: UXT-V2 inhibits P53 by promoting ubiquitin degradation of P53 through MDMX. Down-regulation of P53 activity leads to selective activation of NF-κB signaling pathway, up-regulation of HIF-1α expression, promotion of glycolysis gene *GLUT-1/3, HK-2, LDHA, and ENO* expression, and promotion of glycolysis. These changes promote cell proliferation. By binding to DNMT3B, UXT-V2 downregulates MEG3 by methylation and thus inhibits the P53 signaling pathway. When P53 is suppressed, apoptosis is inhibited and cell proliferation, migration and invasion are promoted.

### 3.4 UXT and DNA methylation

DNA methylation is an epigenetic process. Cancer often shows overall DNA hypomethylation compared with healthy tissues. Methylation of CpG islands in promoter regions generally suppresses transcription; DNA methylation at CpG sites is the most common epigenetic inhibition of tumor suppressor genes in malignant tumors (60, 61). Regulation of genes involved in apoptosis, mediated by DNA methylation, may be an important mechanism for tumor cells to escape apoptosis, and changes in these related genes can occur in the form of hypomethylation to reactivate anti-apoptotic genes or in the form of hypermethylation to inhibit pro-apoptotic genes (62, 63).

DNA methylation can be catalyzed by the DNMT family of enzymes. In breast cancer cells, UXT-V2 interacts with DNMT3B to downregulate *MEG3* through methylation, and negatively regulates the *MEG3/P53* axis, thereby inhibiting apoptosis and promoting proliferation (22). Enhancer of zeste homologue 2 (EZH2) is a catalytic subunit of histone methyl-transferase and polycomb repressive complex 2 (PRC2), which can alter the expression of downstream target genes through H3K27me3 (64, 65). Subsequent studies have found that UXT promotes the formation of the PRC2 complex through interaction between UXT and EZH2 in the nucleus, thus promoting histone methyltransferase (HMTase) activity of EZH2. UXT inhibits transcription of tumor suppressor gene *homeobox A9 (HOXA9)* and *disabled homolog 2 (DAB2)*-interacting protein (DAB2IP), promoting proliferation, colony formation and migration of renal clear cell carcinoma (13). Meanwhile, UXT is highly expressed in breast cancer and that UXT suppresses RND3 epigenetically by recruiting EZH2 in breast cancer. After UXT knockdown, cell proliferation and metastasis are inhibited (66). This evidence suggests that UXT interacts with EZH2 in tumor cells.

Knockdown of EZH2 or DZNep(EZH2 inhibitor) can induce apoptosis of RKO and HCT116 cells, promote autophagy, inhibit G1/S transition, and increase the number of G1 phase cells (67). Meanwhile EZH2 modulates E2F1-dependent apoptosis through epigenetic regulation of Bcl-2 interacting mediator of cell death (BIM) expression (68). Therefore, EZH2 can regulate cell apoptosis, cell cycle and disease progression, playing a crucial role in the occurrence and development of tumors (64, 69). We speculate that UXT may regulate tumor cell apoptosis or other processes by recruiting EZH2 or stabilizing EZH2 as a chaperone (**Figure 3**).

**Figure 3:** UXT and methylation: HOXD9 acts on the UXT promoter to up-regulate UXT expression. UXT promotes methyltransferase activity with EZH2 in PRC2 and methylates the promoter of the tumor suppressor gene *RND3/HOXA9*. The expression of RND3/HOXA9 is down-regulated and promotes tumor cell proliferation, migration and colony formation.

In conclusion, UXT-V1/V2 may regulate apoptosis *via* multiple mechanisms . In the treatment of tumors, the deletion of pro-apoptotic genes or overexpression of anti-apoptotic genes causes the tumor to inhibit apoptosis. This inhibition leads to resistance to chemotherapy drugs and the development of multidrug resistance. UXT may be a potential diagnostic or therapeutic biomarker.

## 4 UXT and autophagy

Autophagy is a conserved mechanism in various cells, is divided into either non-selective or selective. Non-selective autophagy can be used to break down cellular proteins, lipids, and nucleic acids to maintain intracellular homeostasis when cell nutrition is deficient. In selective autophagy, misfolded and abnormally accumulated proteins can be broken down when the body is exposed to conditions such as hypoxia, oxidative stress, pathogen infection, and radiation (70, 71). Autophagy is involved in cell death and survival in cancers, neurodegenerative diseases, and metabolic disorders (72, 73). The NCCD classifies autophagy-dependent RCD as autophagy-dependent cell death (34). During cell death, autophagy can also activate apoptosis, ferroptosis, necrotic apoptosis, and other RCD modes through molecular pathways such as TRAIL and ferritin (70, 74–76). Notably, autophagy-dependent cell death should not be confused with other modes of RCD caused by autophagy (34, 73, 77). Mutations in genes associated with autophagy are associated with many human diseases, and the search for new therapeutic targets in the autophagy pathway has great potential (78).

UXT plays a role in late endosome/autophagosome–lysosome fusion events. Downregulation of UXT leads to an increase in the binding of tumor susceptibility gene 101(TSG101) vesicles to lysosomes, increases autophagy flux, and promotes the degradation of centrosomal protein of 55 kDa (CEP55) when TSG101 is overexpressed (26). In addition, UXT interacts with the mTOR protein, an essential negative regulator of autophagy. In mammals, the mTOR protein participates in the formation of mTOR complex 1 (mTORC1) and mTOR complex 2 (mTORC2) (79). mTORC1 limits the autophagic decomposition of cell components, inhibits the formation of autophagosomes, and plays a role in both the early and late stages of autophagy (80). Conversely, mTORC2 participates in the regulation of apoptosis and glucose homeostasis by interacting with protein kinase B (AKT). In the mouse photosensitive cell line 661W, after the conditional knockout of UXT, the decrease in mTOR activity promoted a significant increase in autophagy-related genes and the inhibition of autophagy-negative regulation genes, accompanied by a decrease in sequestosome 1 (SQSTM1) levels and an increase in microtubule-associated protein light chain (LC3)-II levels. Significant activation of autophagy increases the expression of pro-apoptotic genes and decreases that of anti-apoptotic genes (27). Eventually, photoreceptor apoptosis and the downregulation of retinal pigmentation-related genes lead to severe retinal degeneration and retinal dysfunction. Therefore, UXT plays a key role in promoting mTOR activity to prevent retinal degeneration.

In selective autophagy, P62 acts as a ubiquitin-dependent autophagy-selective receptor that binds to misfolded proteins and mediates protein autophagy degradation (71). P62 may also interact with TRAF6 and activate the NF-κB signaling pathway *via* the P62-TRAF6-NF-κB axis. Additionally, P62 is associated with exogenous apoptosis and autophagy, which can control cell death or survival (81). This hypothesis was partially supported by a subsequent study. UXT-V2 interacts with the autophagy receptor P62 through the LIM protein-binding (LB) domain and acts as an autophagy adapter for P62, regulating P62-mediated selective autophagy (24). Notably, UXT-V2 may act in the form of oligomers. In addition, UXT-V2 specifically interacts with STING1 and selectively autophagy degrades STING1 by promoting the interaction of P62 with STING1 (25). Therefore, UXT-V2 is involved in the selective autophagy degradation of proteins *via* P62 (**Figure 4**).

**Figure 4:** UXT and autophagy: UXT-V2 can be combined with TSG101. When UXT-V2 is down-regulated, it promotes the binding of TSG101-containing vesicles to lysosomes and promotes the degradation of CEP55. At the same time, the expression of LC3-II was up-regulated. UXT interact with mTOR, When UXT-V2 is down-regulated, autophagy promotes genetic *Atg4b/Uvrag/Wipi1/Vps11/Atg9b/Tfeb/Vps18* expression are suppressed. And then inhibit autophagy. P62 can form a strip α-helical structure. UXT-V2 promotes the interweaving of P62 into a network, increases the binding sites of P62 and LC3, and promotes the autophagy degradation of SOD1 aggregates and STING1.

Excessive activation of autophagy can lead to ferroptosis (82). This unique cell death pattern is driven by iron-dependent phospholipid peroxidation and is regulated by iron therapy, redox homeostasis, mitochondrial activity, and lipid and glucose metabolism in the cell, with many signaling pathways (83). Ferroptosis is a mode of cell death involved in the progression of tumors and degenerative diseases. After the activation of autophagy, ferritin in fibroblasts and cancer cells can be degraded to promote ferroptosis (75).

Nuclear factor erythroid 2-related factor 2 (NRF2) and its main negative regulator Kelch-like ECH-associated protein 1 (KEAP1) are essential for maintaining redox, metabolism, and protein homeostasis and regulating inflammation (84). The P62-NRF2 pathway is strongly associated with ferroptosis. In hepatocellular carcinoma, the degradation of KEAP1 mediated by P62 assists the activation of NAD(P)H quinone dehydrogenase 1 (NQO1), heme oxygenase 1 (HO1), and ferritin heavy chain 1 (FTH1) down-stream of NRF2. These downstream genes confer resistance to ferroptosis by altering iron metabolism and lipid peroxidation. Inhibition of NRF2 activation makes HCC cells more susceptible to ferroptosis both *in vitro* and *in vivo*. Thus, NRF2 activation inhibited ferroptosis in liver cancer cells (85). When autophagy is inhibited, the P62-KEAP1-NRF2 pathway protects HepG2 cells from alcohol-induced ferroptosis (86). The P62-KEAP1-NRF2 pathway also protects neuroblastoma cells from 6-OHDA-induced ferroptosis by activating HO1. Targeting the P62-KEAP1-NRF2 signaling pathway provides new insights into the treatment of Parkinson’s disease (87). Similar studies have been performed on lung epithelial cells and neurons in spinal cord injury (88, 89). Thus, we speculate that UXT may regulate ferroptosis in cancer and neurodegenerative diseases through the P62-KEAP1-NRF2 signaling pathway.

Autophagy is a continuous and complex dynamic process, and the effects of UXT regulation on autophagy are not fully understood. Based on the results of previous studies, we believe that UXT may have a dual effect on autophagy regulation. When the expression of UXT is reduced, autophagy can be promoted by reducing the activity of mTOR or promoting the formation of autophagic lysosomes. In contrast, UXT can promote P62-mediated selective autophagy. Based on this, we discussed the possibility that UXT is involved in the regulation of ferroptosis *via* P62. UXT belongs to one of the subunits of pre-folded protein analogs and can act in the form of oligomers. Therefore, studies investigating the mechanism of UXT should consider that in addition to UXT alone, UXT may assist autophagy-related proteins in maintaining the correct protein conformation and function as chaperones, which then regulate autophagy.

## 5 UXT and immunity

The immune system is a complex and effective defense system of the human body. When bacteria, viruses, damaged cells, or tumor cells are used as antigens to stimulate immune cells, they can trigger innate or adaptive immune responses that maintain immune balance in the body. The immune system can also respond to the body’s own components, and the destruction of cells or tissues can lead to autoimmune diseases. In the treatment of tumors, the weak immunogenicity of the tumor itself, inhibition of tumor cell apoptosis, tumor immunosuppressive cells in the tumor microenvironment (TME), and other factors can lead to tumor cells escaping immune surveillance. Cancer immunotherapy is to reactivate tumor immunity by improving immune cell function, immune checkpoint inhibitors, adoptive cell therapy and other methods (90). Thus, immunotherapy for tumors is considered promising.

MAVS is an antiviral protein complex in the mitochondria. Viral infection can activate the MAVS-TNFR3 signaling axis in the mitochondria. As a component of the MAVS signaling body in the mitochondria, UXT-V1 binds to TRAF3 *via* the N-terminal TRAF binding motif, mediates innate antiviral responses. When UXT-V1 is knockdown, the translocation of TRAF3/TRADD to the mitochondria is significantly blocked, which inhibits retinoic acid-inducible gene-I (RIG-I)-mediated IFN-β, IL-8, and interferon-stimulated gene factor 54 (ISG54). Therefore, UXT-V1 is critical for the virus-induced activation of NF-κB and IRF3 and is a positive regulator (28). UXT-V2 is phosphorylated by BGLF4 at the Thr3 site, which blocks the interaction between UXT-V2 and P65; this inhibits the transactivation of NF-κB, effectively weakening the immune response of host cells in the antiviral response, and facilitating the replication process of the virus (29).Therefore, UXT-V2 and UXT-V1 can regulate the innate immune response during viral infection. However, the two mechanisms differ. Since UXT-V1 is primarily present in the cytoplasm, it functions through the mitochondrial MAVS complex. UXT-V2 mainly exists in the nucleus and can act as a component of the NF-κB signal enhanceosome (**Figure 5**).

**Figure 5:** UXT promotes immune response: ​As one of the components of the MAVS signalosome, UXT-V1 promotes the nuclear translocation of IRF3 and NF-κB by binding to TRAF3, thus promoting innate immune response. UXT-V2 can be phosphorylated by BGLF4, disrupting its NF-κB enhanceosome function.

UXT has been shown to be an important negative regulator of type I IFN signaling. UXT also modulates the suppressive phenotype of Treg. Thus UXT may promote immunosuppression. Systemic lupus erythematosus(SLE) is an autoimmune disease characterized by overexpression of type I IFNs and ISGs. After DNA mimics or cGAMP stimulation, UXT specifically binds to STING1 and promotes the binding of STING1 to P62. UXT reduces the production of type I IFN by selectively degrading STING1 (25). UXT can negatively regulate the cGAS-STING1 pathway. Notably, the authors performed a large-scale gene expression profiling using leukocytes and peripheral blood mononuclear cells from 1211 SLE patients and 139 healthy donors and confirmed that UXT expression was significantly impaired in SLE patients (25). ​This provides evidence for the involvement of UXT in the SLE process. In the TME, Tregs participate in the formation of the tumor inhibition microenvironment. Tregs are a subset of T cells and a T cell subtype with immunosuppressive effects primarily involved in adaptive immune responses and play an important role in maintaining immune self-tolerance and immune homeostasis (91). FOXP3, a member of the fox family, is a major regulator of Treg phenotype and immune-suppressive function (92). UXT-V2 is expressed in Tregs, traditional T (ConvT) cells, and B cells in blood samples from healthy volunteers. UXT-V2 directly regulates FOXP3 in Tregs and promotes its transcription by interacting with the proline-rich domain at the N-terminus of FOXP3 in the nucleus (93). Thus, UXT can regulate the inhibitory phenotype of Tregs by promoting the expression of FOXP3.

Based on these previous findings, we conclude that UXT may have a dual effect on innate immunity. UXT-V1/V2 modulates the NF-κB signaling pathway in different ways and modulates innate immunity. In contrast, UXT promotes selective autophagy and inhibits type I IFN production *via* cGAS-STING1 and adaptive immune responses by promoting Treg function. This could be related to the differences between cells and diseases, as well as the different mechanisms of UXT. As there are very few studies on UXT, we cannot rule out the possibility of their simultaneous occurrence. This requires interpretation from a more comprehensive perspective (**Figure 6**).

**Figure 6:** UXT inhibits the immune response: ​UXT-V2 negatively modulates the cGAS-STING1 signaling pathway by promoting the autophagy degradation of STING1 mediated by P62. These changes lead to a down-regulation of the type I IFN expression.

Immunogenic cell death (ICD) refers to the activation of the host adaptive immune response by substances released after cell death as endogenous (such as cell components) or exogenous (such as viruses) antigens after the stimulation of viral infection, chemotherapy drugs, and radiotherapy (34, 94). These changes cause cell death, and is different from traditional apoptosis. ICD stimulates the host immune system and enhances the immune response induced by immunotherapy (95, 96). Therefore, successful induction of ICD is important for improving current oncological treatment outcomes (97). Depending on the complexity of the immunosuppressive TME and the low immunogenicity of tumor cells, the sensitivity to tumor chemotherapy can be reduced, resulting in limited clinical efficacy. Therefore, a more efficient treatment strategy is urgently needed (98). The immune response is the basis of ICD. Manipulating the patient’s immune system to activate the host immune response to the pathogenesis of cancer is a promising strategy. This may provide possible intervention measures to improve tumor metastasis and drug resistance (99).

Several studies have shown that STING1 is effectively activated by various factors that promote ICD in colon cancer and neuroblastoma cells (100, 101). Type I IFN, a cytokine released when tumor cells die, initiates adaptive immunity during ICD and promotes the maturation of antigen-presenting cells (94, 102). Type I IFN directly promotes DC maturation and links innate and adaptive immunities (103). As a subunit of the pre-folded protein family, UXT participates in tumor cell antigen exposure and antigen presentation, thereby affecting the number of tumor-infiltrating immune cells (TIICs) (104). In addition, Tregs recognize autologous and non-autologous antigens, including tumor antigens, and down-regulate dendritic cell function through CTLA-4, granulozyme/perforin, and IL-10, thereby disabling T cell activation responses and inducing immunosuppression and immune tolerance (105). Immune tolerance can hinder effective tumor immunity. Numerous Tregs infiltrate the human liver, lung, pancreas, and other tumors (106–108). Changes in tumor infiltration are critical to the outcome of antitumor drug therapy, and an increase in the proportion of Tregs indicates a poor treatment response (109). The removal of Tregs can reduce tumor immune tolerance, thereby improving the efficacy of tumor immunotherapy and increasing the risk of autoimmune diseases (110). Therefore, effective tumor immunity can also be obtained through systemic or local disruption of immune tolerance. EZH2 has been shown to maintain the immunosuppressive function of Tregs by modulating the transcription of Tregs cells (111). As described above, UXT interacts with EZH2 in the nucleus to promote the activity of the methyltransferase in which EZH2 is involved. Interestingly, blocking the function of EZH2 in Treg selectively breaks tolerance in the TME without inducing systemic autoimmune toxicity (112). Therefore, knocking down UXT to inhibit Tregs may create a favorable immune basis for the occurrence of ICD.

UXT may be involved in the regulation of ICD in two ways. On the one hand, UXT may enhance the immune response by modulating the expression of type I IFN and immunosuppressive cells, while on the other hand, UXT may also regulate antigen exposure and presentation and promote the maturation of antigen-presenting cells. UXT is down-regulated to reduce EZH2 recruitment, thereby improving the autoimmune toxicity caused by inhibition of Treg cells.

As previously indicated, UXT-V2 can up-regulate the expression of glycolysis-related genes and promote tumor glycolysis (5). Hypoxia is one of the characteristics of the TME in solid tumors. According to the Warburg effect, tumor cells prefer glycolysis for their energy supply even under aerobic conditions. A large amount of pyruvate is produced during glycolysis and that energy supply and is then converted into lactic acid by lactate dehydrogenase (LDH). Lactic acid is one of the main contributors to an acidic TME. In acidic TMEs, many tumor cells, including breast cancer cells, experience immuno-suppression (113). Lactic acid promotes the survival of melanoma cells in acidic TME (114). In addition, lactic acid plays an immunosuppressive role in the TME, increases tumor cell survival and promotes tumor immune escape (115).

Therefore, inhibition of glycolysis reduces the concentration of lactate to reshape the TME and enhance anti-tumor immunity (116). Several studies have shown that the inhibition of glycolysis promotes ICD induction in hepatocellular carcinoma (117). Thus, we speculate that targeting UXT to improve tumor metabolic reprogramming promotes ICD in tumor cells. Notably, lactic acid promotes the activity and recruitment of Tregs, which reduces the immune response of the cancer cells (118). Tregs express the lactate transporter monocarboxylate transporter 1 (MCT1) and transport lactate as a metabolic fuel (119) (**Figure 7**).

**Figure 7:** UXT regulates the tumor microenvironment: ​UXT-V2 promotes glycolysis by selectively activating the NF-κB signaling pathway by inhibiting the P53 signaling pathway. Glycolysis is promoted to increase lactate production and to acidify the TME. When UXT-V2 expression is up-regulated in Tregs, FOXP3 mRNA and protein levels are also up-regulated. UXT-V2 can also help maintain the inhibitory phenotype of Treg by binding to FoxP3 and stabilizing FOXP3 binding to *IL-2/CTLA-4/CD25* promoters.

In summary, UXT can promote the function of Tregs, and, conversely, glycolysis in tumor tissues. These two factors may contribute to each other by exacerbating immunosuppression, immune escape, and promoting tumor progression. Therefore, targeted UXT may improve therapeutic effects by improving tumor cell metabolism in the TME. In addition, targeted UXT may promote ICD by improving tumor antigenicity, improving antigen presentation, and enhancing the immune response.

## 6 UXT and neurodegenerative diseases

ALS is a progressive neurodegenerative disease characterized by degeneration of motor neurons in the brain and spinal cord, accompanied by progressive muscle weakness. The ALS2 protein encoded by the *ALS2* gene is closely related to diseases of the nervous system, including ALS. The accumulation of abnormal proteins caused by mutations in ALS2 or other factors can cause many clinical symptoms or different diseases (120, 121). ALS results in paralysis and death within 2–5 years of onset.

ALS is a disease involving multiple systems and factors. Although the etiology and pathogenesis of ALS are not fully understood, research has shown that inflammatory responses in the peripheral and central nervous systems contribute to the injury of motor neurons and promote disease progression. The pathological processes of ALS2 involve endoplasmic reticulum stress, oxidative stress, neuroinflammation, and axonal transport dysfunction, and the study of the relationship between the structure and function of the ALS2 protein and the study of interacting proteins or chaperones will provide novel insights into the molecular pathogenesis of ALS (122) (**Figure 8**).

**Figure 8:** UXT regulates the degradation of SOD1 protein aggregates in ALS: UXT-V2 promotes autophagy degradation of P62 - mediated SOD1 protein aggregates. UXT-V2 promotes endolysosomal trafficking of SOD1 protein aggregates by binding to ALS2.

​Several researchers have found that UXT interacts directly with ALS2 and is co-localized in the cytoplasm (123, 124). The UXT-V2 isoform protein specifically interacts with ALS2 *in vitro* and *in vivo* through its DH/PH region. In addition, UXT-V2 and ALS2 were colocalized in the cytoplasm of Neuro2a cells. Interestingly, their transcription appears to be synchronized throughout the cell cycle, with G0/G1 being the highest expression phase for both genes (125). Previous studies have found that overexpression of ALS2 triggers the Rac1/phosphatidylinositol 3-kinase/Akt3 anti-apoptotic pathway, thus inhibiting the toxicity of superoxide dismutase type 1 (SOD1) (126). The central nervous system is rich in SOD1, which accounts for approximately 1% of brain proteins. Mutated SOD1 exhibits definite neurotoxicity; SOD1 mutations are prone to form aggregates due to misfolding. SOD1 is associated with ALS. In addition, ALS2 has a protective effect on SOD1 and can bind to mutant SOD1 to inhibit its toxicity. As one of the subunits of a pre-folded protein analog, UXT may help to maintain the proper folding of mutant SOD1 close to the DH/PH region of ALS2 to some extent, thus assisting in its protective effect on SOD1.

Mutated P62 causes motor neuron degeneration in mice and zebrafish ALS models (127, 128). The interaction between UXT and the autophagy receptor P62 can prevent protein toxicity in neurons by facilitating autophagy degradation of protein polymers (24). Thus, UXT may play a protective role in ALS by acting as a chaperone protein, helping the protein maintain its normal conformation, or promoting selective autophagy to weaken endoplasmic reticulum stress caused by abnormal protein accumulation.

ALS-associated mutations enhance the accumulation of TAR DNA-binding protein 43 (TDP-43) in the cytoplasm and mitochondria (129). Accumulation of TDP-43 in the cytoplasm is a marker of ALS and has been linked to neuroinflammatory cytokines in patients with ALS. NF-κB and type I IFN can upregulate relevant inflammatory factors and promote disease progression in ALS. One study found that TDP-43 leads to the mitochondrial DNA (mtDNA) entering the cytoplasm after entering the mitochondria, activating IRF3, and upregulating NF-κB activity by activating the cGAS-STING signaling pathway. Remarkably, researchers have been able to delay neurodegeneration by downregulating the STING signal, demonstrating the potential of targeting this pathway (130). In addition, STING can degrade the autolysosome pathway in the bone marrow cells. Blocking STING suppresses the overactive type I interferon response and inflammation in immune cells caused by a C9orf72 deficiency (131). Therefore, STING is an exciting potential target for ALS transformation therapy (132). UXT-V2 degrades STING through selective autophagy, negatively regulates the cGAS-STING1 signaling pathway, and reduces type I IFN production (25). We speculate that UXT may play a neuroprotective role in ALS by promoting autophagic degradation of STING and negatively regulating type I IFN.

Compared with the control group, one study found that the number of T cell subsets in patients with ALS significantly increased CD8 cytotoxic T cells and natural killer (NK) T cells, while Tregs significantly decreased. Tregs are also negatively correlated with disease progression. This indicates that patients with ALS exhibit systemic immune activation (133). A prospective multicenter human and animal experiment showed that Treg expansion was negatively correlated with disease progression rate and positively correlated with survival time. In addition, the expansion of Tregs was associated with a decrease in somatic cell size of motor neurons in SOD1 mutant mice, significant suppression of astrocyte and microglial immunoreactivity, and increased expression of neurotrophic factor genes in the spinal cord and peripheral nerves. Thus, Tregs have a protective effect on the nerves and may also inhibit toxic neuroinflammation in the central nervous system. The strategy of peripheral enhancement and neuroprotective activity of the Treg group may prove to be therapeutic in patients with ALS (134). Notably, it is generally safe and well-tolerated to inject Tregs into the body in combination with IL-2 subcutaneously after conducting a phase I uncontrolled clinical trial. This slows the progression of both the early and late stages of the disease (135). In subsequent randomized control trial and open-label extension, it was found that Treg/IL-2 treatment was safe, well-tolerated, and had a high Treg inhibition function (136) (**Figure 9**).

**Figure 9:** UXT regulates neuroinflammation in ALS: UXT-V2 down regulates the expression of type I IFN by autophagy degradation of STING1 mediated by P62. UXT-V2 promoted the inhibitory phenotype of Tregs by binding to FOXP3. Together, they improve neuroinflammation in neurodegenerative diseases.

Therefore, the protective effect of Tregs on nerves in ALS has been preliminarily proven both theoretically and clinically. As mentioned earlier, UXT regulates Tregs through Foxp3. When UXT was overexpressed in Tregs, the binding of Foxp3 to *IL-2, CTLA-4, and CD25* increased. We speculate that UXT plays a neuroprotective role in ALS by negatively regulating the cGAS-STING1 signaling pathway and positively regulating the nuclear localization and stability of the Foxp3 protein, thereby inhibiting the progress of neuroinflammation in ALS.

The interaction between UXT and Down syndrome (DS) critical region gene 1 (DSCR1) on human chromosome 21 has been previously confirmed *in vitro* (137).

DSCR1 is also called calcineurin (RCAN) in subsequent studies and is believed to be involved in the pathogenesis of DS (138). RCAN homologues are upregulated in Alzheimer’s disease, myocardial hypertrophy, diabetes, and degenerative neuropathy, as well as in external stressors (such as reactive oxygen species, Ca^2+^, β-amyloid, and hormone changes) (139). Research on whether and how UXT may play a role in DS has not progressed.

## 7 Conclusions and future directions

Chemotherapy and radiotherapy play an irreplaceable role in tumor treatment. However, chemoresistance or multidrug resistance is a difficult problem that has plagued human beings for many years. UXT-V1 regulates TNF, induces the formation of the TNFR1 trimer, inhibits the recruitment of TNFR1 signal complex, and inhibits apoptosis. UXT-V2 inhibits cell apoptosis by promoting the expression of anti-apoptotic genes downstream of NF-κB and by epigenetic inhibition of the P53 signaling pathway. UXT-V2 interacts with the mitochondria and SARM to promote apoptosis. When the expression of UXT is reduced, it can promote autophagy by promoting the fusion of vesicles and lysosomes. It can also promote autophagy and cause photoreceptor apoptosis by interacting with mTOR. In addition, UXT interacts with P62 to promote selective autophagy mediated by P62. Thus, UXT can regulate apoptosis and autophagy in various ways and regulate the regulatory death of tumor cells. This suggests the possibility of UXT involvement in the diagnosis and treatment of tumors and in alleviating drug resistance to chemotherapy. The effect of the P62-KEAP1-NRF2 axis on ferroptosis in tumor cells has been previously reported; therefore, we discussed the possibility of UXT involvement in P62-mediated ferroptosis. We hope to further deepen the understanding of the effect of UXT on tumors from the perspective of regulatory cell death.

With the application of immune checkpoint inhibitors, CAR-T cells, adoptive immunotherapy, and other therapies, tumor immunotherapy is widely considered to be promising. In recent years, there has been a gradual increase in the study of UXT in the immunological community. UXT-V1 inhibits type I IFN expression through the cGAS-STING signaling pathway and participates in innate immune response. ​The cGAS-STING signaling pathway has a strong immune surveillance effect. ​Activation of the STING promotes a variety of anti-tumor effects, including T cell activation, DC maturation, and accelerated cancer cell death. ​STING also modulates inflammation and type I IFN induced disease progression in ALS and SLE. ​UXT interacts with the Foxp3 to regulate the inhibitory phenotype of Treg and participate in the adaptive immune response. Meanwhile UXT may also regulate gene transcription in Treg through EZH2.Treg is a type of CD4^+^T cell that is immunosuppressive. This effect is seen in both tumors and ALS. ​UXT can promote autophagy degradation of STING and inhibitory phenotypes of Treg. ​This provides a clue to the immunosuppressive effects of UXT in diseases including tumors and neurodegenerative diseases. ​UXT can also up-regulate the expression of glycolytic genes through a crosstalk between the P53 and NF-κB pathways. ​This not only enhances tumor cell proliferation and anti-apoptotic advantage, but also promotes lactate production in TME. ​Lactate promotes the formation of the acid TME and acts as a fuel for Treg to maintain the immunosuppressive function of Treg. ​Therefore, UXT may have immunosuppressive function on the one hand and metabolic regulation on the other. ​Through the connection of these two aspects, it is possible not only to promote tumor cell survival, but also to cause more severe immunosuppression. Importantly, RIG-I-mediated expression of IFN, IL-8 and ISG54 can be suppressed by MAVS when UXT-V1 is down-regulated. Phosphorylation of UXT-V2 blocks the activation of NF-κB and attenuates the host’s antiviral immune response.

The study of UXT in cell death and immunity is still in its infancy; therefore, the available data are limited, with some key questions requiring further explanation. First, in a specific disease or mechanism study, we must identify the isoforms and action forms of UXT. There are two isoforms of UXT with different cell distributions. Although UXT-V1 and UXT-V2 are distributed in the nucleus, cytoplasm and mitochondria, UXT-V1 is mostly found in the cytoplasm, while UXT-V2 in the nucleus. At the same time, except for the monomer form, the structure of UXT has the ability to form a hexamer. Second, there have been few studies of UXT interaction targets, mechanisms and related diseases. As a target discovered more than 20 years ago, UXT-related malignancies are more concentrated in breast and prostate cancers, where it is believed to regulate tumor progression and affect tumor prognosis. The mechanisms of UXT mainly involve NF-κB, P53, methylation, autophagy and androgen receptors. Therefore, research on other diseases and their mechanisms remains warranted.

## Author contributions

PH, YT and XF contributed to conception and design of the study. PH and SM drafted and revised the manuscript. PH, SM, ZW and JX contributed to the production and modification of images. YT made critical revisions to important parts of the manuscript. All authors contributed to manuscript, and approved the submitted version.
